This article has been retracted.

# Analysis of Inducing Factors of Chronic Pulmonary Heart Disease Caused by Chronic Obstructive Pulmonary Disease at High Altitude through Epidemiological Investigation under Intelligent Medicine and Big Data

**DOI:** 10.1155/2022/2612074

**Published:** 2022-01-12

**Authors:** Jiong Huang, Fulin Dang

**Affiliations:** ^1^Emergency Department, Huangyuan County People's Hospital, Xining 812100, China; ^2^Huangyuan County People's Hospital, Xining 810000, China

## Abstract

This study explores the risk factors of chronic pulmonary heart disease (CPHD) induced by plateau chronic obstructive pulmonary disease (COPD) based on intelligent medical treatment and big data of electrocardiogram (ECG) signal. Based on GPU, a wavelet algorithm is introduced to extract features of ECG signal, and it was combined with generalized regression neural network (GRNN) to improve classification accuracy. From June 2018 to December 2020, 10,185 patients diagnosed with COPD in the plateau area by pulmonary function testing, ECG, and chest X-ray at X Hospital are taken as the research objects to evaluate the distribution of CPHD incidence at different ages and altitudes. The running time of GTX780Ti is about 15 times shorter than that of CPU. The accuracy of N detection based on the GPU-accelerated neural network model reached 98.06%. Accuracy (Acc), sensitivity (Se), specificity (Sp), and positive rate (PR) of V were 99.03%, 89.17%, 98.92%, and 93.18%, respectively. The Acc, Se, Sp, and PR of S were 99.54%, 86.22%, 99.74%, and 92.56%, respectively. The GRNN classification accuracy was up to 98%. 19% of COPD patients were diagnosed with CPHD, including 1,409 males (72.82%) and 526 females (36.24%). The highest prevalence of CPHD was 64.60% when the altitude was 1,900–2,499 m, and the prevalence was only 2.43% when the altitude was ≥3,500 m. The highest prevalence of CPHD was 63.77% at the age of 61–70 years, and the lowest prevalence at the age of 15∼20 years was only 0.26%. Therefore, the GPU-based neural network model improved the classification accuracy of ECG signals. Age and altitude were risk factors for CPHD induced by high-altitude COPD, which provided a reference for the prevention, diagnosis, and treatment of CPHD in high-altitude areas.

## 1. Introduction

Chronic obstructive pulmonary disease (COPD) is a common persistent respiratory disease. In recent years, with the development of economy, the prevalence and mortality of COPD have increased year by year. About three million people die of COPD every year in the world [1]. It is estimated that more than 4.5 million people worldwide will die from COPD in 2030 [2]. As the prevalence of COPD increases, the prevalence of chronic pulmonary heart disease (CPHD) also increases. Current research results showed that COPD is the main cause of CPHD, accounting for about 87% of the prevalence of CPHD [3]. However, the current prevalence of COPD and CPHD in plateau areas and the influencing factors are still unclear, and further research is needed.

With the development of Internet cloud computing and other information technologies, smart healthcare and big data are widely utilized in transportation, banking, medical, and education industries [4–6]. Intelligent medical big data is a collection of data information in the medical industry. In the actual application process, intelligent medical big data has disadvantages such as a variety of data types, complex relationships, and explosive growth [7]. In particular, the problem of computational burden is obvious, and it often takes hours or even days to analyze big medical data [8]. In response to this problem, researchers proposed that parallel processing of existing data can save processing time and increase the efficiency of medical data analysis [9]. However, this method will produce corresponding message transmission overhead. Fernandez et al. designed molecular dynamics parallel algorithms based on GPU, and its computational efficiency increased by about 10 times [10]. Paulose et al. utilized artificial neural network algorithms based on CPU to improve the accuracy of data mining [11]. However, there are currently few studies on the combination of GPU and neural network algorithms to improve the efficiency of medical big data analysis while improving accuracy.

To sum up, GPU and neural network algorithms have significant advantages in processing medical big data, but there is little research on combining the two in the medical big data processing. Therefore, patients with COPD in the plateau area were the research subjects. A neural network model method based on GPU acceleration was established and applied to extract electrocardiogram (ECG) signals and QRS wave positioning. Then, the inducing factors of high-altitude COPD to CPHD were analyzed to provide a reference for the prevention, diagnosis, and treatment of CPHD in high-altitude areas.

## 2. Materials and Methods

### 2.1. Research Objects

A total of 10,185 patients diagnosed with COPD in high-altitude areas by pulmonary function test, electrocardiogram, and chest X-ray in X Hospital from June 2018 to December 2020 were selected as the research subjects. There were 5,349 males and 4,836 females. The patients's age ranged from 15 to 85 years, with a mean age of 63.92 ± 4.46 years. Inclusion criteria for this study were as follows: (i) all patients had COPD in the high-altitude area; (ii) acute exacerbation of COPD was defined as an acute exacerbation of cough, sputum, asthma, and increased sputum volume, purulent or mucous purulent, accompanied by fever and greatly increased inflammation. Exclusion criteria were as follows: (i) patients with bronchiolitis obliterans, tuberculosis, pulmonary interstitial fibrosis, bronchiectasis, and bronchial asthma; (ii) congenital heart disease, coronary heart disease, valvular heart disease, and cardiomyopathy; pulmonary arterial hypertension, left heart disease, chronic thromboembolism, and other diseases causing pulmonary hypertension; (iii) patients complicated with a blood disease, liver disease, kidney disease, and tumor. The experimental procedure of this study had been approved by the Ethics Committee of the Hospital, and all the subjects included in the study had signed the informed consent.

### 2.2. ECG Signal Processing Method Based on GPU Acceleration

The characteristics of the ECG signal are extracted by calibrating the PQRST wave of the ECG. Wavelet transform is an efficient method for extracting QRS waves from ECG, but the algorithm takes a long time in the actual application process [12]. Therefore, GPU parallel processing was adopted for the calibrated PQRST wave to increase its computational efficiency. For the initial ECG signal data, the CPU was employed to read the relevant data and then input it to the GPU. After processing using the wavelet transform and Mallat algorithm, the QRS wave is calibrated to obtain the characteristic value of the ECG signal, and finally, the characteristic value is output to the CPU. The ECG signal feature extraction process based on GPU acceleration is shown in Figure 1.

The ECG signal should be preprocessed for power frequency interference, baseline drift, myoelectric interference, and motion artifacts to obtain an effective QRS wave. The wavelet transform method was utilized to extract QRS waves. After the basic wavelet was translated and stretched, the calculation method of the wavelet base was obtained.

(1) $$\begin{array}{c} \varphi_{a,\tau }\left(\text{t}\right)=\frac{1}{\sqrt{a}}\varphi \left(\frac{t-\tau }{a}\right), \end{array}$$

where *a* is the expansion factor, *τ* is the translation factor, and *t* is the time.

It is assumed that *φ*(t) is a basic wavelet and *φ*_*a*,*τ*_(*t*) is a continuous wavelet basis function; the continuous wavelet transforms for any wavelet *f*(*t*) are expressed as follows:

(2) $$\begin{array}{c} Wf\left(a,\tau \right)=\langle f\left(t\right),\varphi_{a,\tau }\left(t\right)\rangle =\frac{1}{\sqrt{a}}\int_{-\infty }^{+\infty }f\left(t\right)\varphi \left(\frac{t-\tau }{a}\right)dt\;. \end{array}$$

The dyadic wavelet transform is a semidiscrete wavelet transform. The scale factor is binary-discrete, while the displacement factor keeps changing continuously; that is, *a*=2^*j*^, *j* ∈ *Z*, and *τ* ∈ *R* [13]. Then, the continuous wavelet basis function is expressed as $\varphi_{2^{j},\tau }\left(t\right)=1/\sqrt{2^{j}}\varphi \left(t-\tau /2^{j}\right)$, and its corresponding wavelet transform is expressed as follows:

(3) $$\begin{array}{c} Wf\left(2^{j},\tau \right)=\frac{1}{\sqrt{2^{j}}}\int_{-\infty }^{+\infty }f\left(t\right)\varphi \left(\frac{t-\tau }{2^{j}}\right)dt\;. \end{array}$$

If the continuous wavelet transform exists, *φ*(*t*) must satisfy *A* ≤ ∑_*j*∈*Z*_|*φ*(2^*j*^*a*)|^2^ ≤ *B*, where *A* and *B* are constants and satisfy the condition 0 < *A* ≤ *B* < *∞*.

Mallat algorithm has important significance in wavelet multiresolution analysis [14, 15]. The two-scale equation of the Mallat algorithm is expressed as follows:

(4) $$\begin{array}{c} \phi \left(t\right)=\sum_{n}h_{0}\left(n\right)\phi_{-1,n}\left(t\right)=\sqrt{2}\sum_{n}h_{0}\left(n\right)\phi \left(2t-n\right),\\ \varphi \left(t\right)=\sum_{n}h_{1}\left(n\right)\phi_{-1,n}\left(t\right)=\sqrt{2}\sum_{n}h_{1}\left(n\right)\phi \left(2t-n\right), \end{array}$$

where *h*_0_(*n*) is the coefficient of the low-pass filter and *h*_1_ is the coefficient of the bandpass filter.

The following equation is obtained by stretching and shifting time:

(5) $$\begin{array}{c} \phi \left(2^{-j}t-k\right)=\sqrt{2}\sum_{n}h_{0}\left(n\right)\phi \left(2^{-j+1}t-2k-n\right). \end{array}$$

*m*=2*k*+*n*; then, there is the following equation:

(6) $$\begin{array}{c} \phi \left(2^{-j}t-k\right)=\sqrt{2}\sum_{m}h_{0}\left(m-2k\right)\phi \left(2^{-j+1}t-m\right). \end{array}$$

According to multiresolution analysis, the following equation is defined:

(7) $$\begin{array}{c} V_{j-1}=\underset{k}{\text{span}}\left\{2^{\left(-j+1\right)/2}\phi \left(2^{-j+1}t-k\right)\right\}. \end{array}$$

Then, the expansion of any *f*(*t*) in space *V*_*j*−1_ is expressed as follows:

(8) $$\begin{array}{c} f\left(t\right)=\sum_{k}c_{j,k}2^{-j/2}\phi \left(2^{-j}t-k\right)+\sum_{k}d_{j,k}2^{-j/2}\varphi \left(2^{-j}t-k\right). \end{array}$$

The expansion coefficients *c*_*j*,*k*_ and *d*_*j*,*k*_ on the *j* scale are expressed as follows:

(9) $$\begin{array}{c} c_{j,k}=\int_{-\infty }^{+\infty }f\left(t\right)2^{-j/2}\phi \left(2^{-j}t-k\right)d,\\ d_{j,k}=\int_{-\infty }^{+\infty }f\left(t\right)2^{-j/2}\varphi \left(2^{-j}t-k\right)d, \end{array}$$

where *j* is the number of scale spaces, *c*_*j*,*k*_ is the scale coefficient, *d*_*j*,*k*_ is the wavelet coefficient, and *V*_*j*−1_ is the scale space. Then, the wave transform coefficient is expressed as follows:

(10) $$\begin{array}{c} c_{j-1,m}=\sum_{k}c_{j,k}h_{0}\left(m-2k\right)+\sum_{k}d_{j,k}h_{1}\left(m-2k\right). \end{array}$$

It is assumed that *θ*(*t*) is a smoothing low-pass function that satisfies the conditions ∫_−*∞*_^+*∞*^*θ*(*t*)*dt*=1, lim*θ*(*t*)=0. Then, the wavelet function is expressed as ∫_−*∞*_^+*∞*^*φ*(*t*)*dt*=0. With *φ*(*t*), the convolutional wavelet transforms of signal *f*(*t*) at the scale of *a* and the displacement of *t* are expressed as follows:

(11) $$\begin{array}{c} Wf\left(a,t\right)=f*\varphi_{a}\left(t\right)=\frac{1}{a}\int_{R}f\left(\tau \right)\varphi \left(\frac{t-\tau }{a}\right)d\tau \;. \end{array}$$

A quadratic spline wavelet function with compact support and first-order vanishing moments was selected, and its Fourier transform is expressed as $\hat{\varphi }\left(\omega \right)=i\omega {\left(\sin\left(\omega /4\right)/\omega /4\right)}^{4}$; then, the low-pass filter and high-pass filter of the shape are expressed as follows:

(12) $$\begin{array}{c} L\left(\omega \right)=e^{i\omega /2}{\left(\cos\frac{\omega }{2}\right)}^{3}=\frac{1}{8}e^{-i\omega }+\frac{3}{8}+\frac{3}{8}e^{i\omega }+\frac{1}{8}e^{2i\omega },\\ H\left(\omega \right)=4ie^{i\omega /2}\left[\sin\frac{\omega }{2}\right]=-2+2e^{i\omega }. \end{array}$$

The discrete Fourier transform of the binary-discrete wavelet transform is as follows:

(13) $$\begin{array}{c} W_{2^{j}}f\left(\omega \right)=\left\{\begin{array}{c} H\left(\omega \right)f\left(\omega \right)\phi \left(\omega \right)\\ H\left(2\omega \right)L\left(\omega \right)f\left(\omega \right)\phi \left(\omega \right)\\ H\left(2^{j-1}\omega \right)L\left(2^{j-1}\omega \right)f\left(\omega \right)\phi \left(\omega \right) \end{array}\right.. \end{array}$$

### 2.3. Neural Network Model Operation Based on GPU Acceleration

Neural network models are widely utilized in model predictions due to their robustness, large-scale parallel processing capabilities, and nonlinear characteristics. The generalized regression neural network (GRNN) calculates the network output by calculating the output value of the model layer and the double-layer neuron. It is assumed that the number of samples is *N*, the sample dimension is *D*, and the number of model layers is *C*. The sample space *X* is expressed as shown in equation (1), where *X*_*i*_ is the *i*-th sample in the dataset.

(14) $$\begin{array}{c} X=\left\{\begin{array}{ccccc} x_{1,1} & x_{1,2} & x_{1,3} & \cdots & x_{1,D}\\ x_{2,1} & x_{2,2} & x_{2,3} & \cdots & x_{2,D}\\ \vdots & \vdots & \vdots & \vdots & \vdots \\ x_{N,1} & x_{N,2} & x_{N,3} & \cdots & x_{N,D} \end{array}\right\}. \end{array}$$

A neuron in the pattern layer corresponds to a learning sample, and the transfer function of the *i*-th learning sample is expressed as follows:

(15) $$\begin{array}{c} f\left(x\right)=\exp\left[-\frac{{\left(x_{in}-x_{i}\right)}^{C}\left(x_{in}-x_{i}\right)}{2\sigma^{2}}\right], \end{array}$$

where *x*_in_ is the network input variable, *x*_*i*_ is the learning sample corresponding to the *i*-th neuron, and *σ* is the smoothing coefficient.

The transfer function in the summation layer that accumulates the outputs of all the model layer neurons is expressed as equation (16). The transfer function of the weighted summation of the outputs of all the model layer neurons is expressed as shown in equation (17), where *y*_*ij*_ is the *j*th element in the *i*-th output sample:

(16) $$\begin{array}{c} S_{a}=\sum_{i=1}^{n}f\left(x\right). \end{array}$$

(17) $$\begin{array}{c} S_{w}=\sum_{i=1}^{n}y_{ij}f\left(x\right). \end{array}$$

The number of neurons in the output layer is the dimension of the output vector in the learning sample, and the calculation method of the prediction result corresponding to the *j*th neuron is expressed as follows:

(18) $$\begin{array}{c} y_{j}=\frac{S_{w}}{S_{a}}. \end{array}$$

According to the ECG results, the corresponding data are read, the numbers of neurons in the input layer, the segmentation dataset, and the smoothing coefficient are set. The obtained data are input into the GPU for ECG signal feature extraction, and the extracted data are output to the CPU. The current evaluation indicator and smoothing coefficient are recorded, and it is judged whether the smoothing coefficient reaches the preset maximum value. If it is not reached, a further smoothing coefficient increment loop is needed. If the smoothing coefficient reaches the preset maximum value, the smoothing coefficient and prediction error value with the best evaluation indicator are selected. Further, whether the number of input neurons reaches the maximum value is judged. If it is not reached, it will enter the neuron coefficient increment loop. If the number of input neurons reaches the maximum, the neuron coefficient and smoothing coefficient with the smallest prediction error are selected to determine the model. The flowchart of the GPU-based GRNN algorithm is shown in Figure 2.

The experimental environment of this study was a home PC, the processor was Intel Core i3-3240, and the main frequency was 3.4 GHz. CUDA C was the programming language, and the debugging environment was Microsoft Visual Studio 2010. The graphics cards utilized were NVIDIA GeForce GTX620, NVIDIA GeForce GTX660, NVIDIA GeForce GTX960, NVIDIA GeForce GTX750Ti, and NVIDIA GeForce GTX780Ti. The comparison of the program parallelization parameters in the article was carried out under GTX620 and GTX660. After the optimal design was obtained, the program was run on GTX960, GTX750Ti, and GTX780Ti for horizontal comparison.

### 2.4. Evaluation of Classification Performance of Neural Network Model Based on GPU Acceleration

According to the *Association for the Advancement of Medical Instrumentation* (AAMI) standard [16], the ECG signal is classified into normal heartbeat (N), supraventricular premature beat (S), ventricular premature beat (V), ventricular fusion heartbeat (F), and unclassified signal (Q). According to the method of Jamshidi et al. [17], accuracy (Acc), sensitivity (Se), specificity (Sp), and positive rate (PR) were calculated to evaluate the classification performance. The calculation methods of Acc, Se, Sp, and PR were as follows:

(19) $$\begin{array}{c} \text{Acc}=\frac{\text{TP}+\text{TN}}{\text{TP}+\text{TN}+\text{FP}+\text{FN}},\\ \text{Se}=\frac{\text{TP}}{\text{TP}+\text{FN}},\\ \text{Sp}=\frac{\text{TN}}{\text{TN}+\text{FP}},\\ \text{PR}=\frac{\text{TP}}{\text{TP}+\text{FP}}, \end{array}$$

where TP is the number of true positives, TN is the number of true negatives, FP is the number of false positives, and FN is the number of false negatives.

### 2.5. Chronic Pulmonary Heart Disease (CPHD) Screening

All COPD patients examined underwent a 12-lead ECG. The results of the examination were completed by the same professional technician and respiratory physician. The diagnosis of CPHD was carried out according to China's CPHD diagnostic standards, and the diagnosis of ECG must have more than two conditions to be diagnosed with CPHD. The diagnostic criteria of CPHD electrocardiogram were as follows: (i) frontal mean electrocardiographic axis (MEA) ≥+90°; (ii) clockwise transposition (V1R/S) ≥1; (iii) severe clockwise transposition (V5R/S) ≤ 1; (iv) pulmonary P wave voltage ≥0.22 mV; (v) pulmonary P wave voltage ≥0.22 mV; (vi) R wave amplitude in lead V1 (Rv1) + S wave amplitude in lead V5 (Sv5) > 1.05mV; (vii) R/Q ≥ 1; (viii) except for myocardial infarction, V1∼3 showing Qs, Qr, and qr.

SPSS 19.0 was employed for data statistics and analysis. Mean ± standard deviation ($\bar{x}\pm s$) was used to express measurement data, and percentage (%) was used to express count data. The data were tested using the *χ*^2^ test.

## 3. Experimental Results

The wavelet filtering method was utilized to extract the features of the electrocardiogram signal, and they were designed to be executed in parallel on GPU and CPU, respectively. The results are shown in Figure 3. Under the same ECG signal processing, as the number of ECG signal groups increased, the program running time showed an increasing trend. The processing time of GPU-based GTX620 and GTX660 graphics cards varied slightly with the increase in the number of ECG signal groups, while the processing time of the CPU increased notably. When ten sets of data were processed at the same time, the GPU processing time was 20.2 times that of the CPU processing. Figure 3 shows the comparison of time-consuming feature extraction of different graphics cards.

The shared memory was utilized to optimize the efficiency of the program in the training process of the classification model to discuss the impact of block allocation to different numbers of threads on the efficiency of program execution. The result is shown in Figure 4. As the number of threads increased, whether shared memory was utilized or not, the running time of the program decreased first and then increased. Moreover, the running time of a program that utilized shared memory was about 4.8 times shorter than that of a program that did not use shared memory. When the number of threads was 192, the running time of the program using shared memory reached the minimum value of 2.64 s. Figure 4 shows the comparison of parallel parameter settings.

The execution efficiency of parallel GRNN based on GPU and CPU design under different training set sizes was compared in Figure 5. As the amount of sample data continued to increase, the running time of different processors showed an obvious upward trend. The processing time of GPU-based GTX620 and GTX660 graphics cards was dramatically less than that of the CPU. When the number of samples was low, the GPU acceleration efficiency was up to 20.05 times faster than the CPU. As the number of samples increased, GPU parallel algorithms were limited by hardware access latency, but their running time was still more than nine times faster than CPU. Figure 5 is the comparison of the execution efficiency of the GRNN algorithm in GPU and CPU.

The operating efficiency of the GRNN algorithm under six different hardware processing was compared in Figure 6. As the number of ECG signals increased, the processing time of different hardware was on the rise. The CPU processing time was the longest, and the GTX780Ti processing time was the shortest. The GTX780Ti running time was about 15 times shorter than that of the CPU. Figure 6 presents the operating efficiency of the GRNN algorithm in different hardware.

The quadratic spline wavelet, Morlet wavelet, and Symlet wavelet were utilized to extract features of the ECG signal, locate the QRS wave, and analyze the results. The quadratic spline wavelet can accurately extract and locate the QRS wave, the Morlet wavelet had missing detection, and the Symlet wavelet had the wrong detection of the P wave.  Figure 7 displays the results of different algorithms to locate QRS waves.

The ECG signal classification results of the neural network model based on GPU acceleration were compared. The highest accuracy of detecting N was 98.06%, and the accuracy of detecting S, V, F, and Q was 91.18%, 89.22%, 84.07%, and 75.46%, respectively.  Figure 8 shows the comparison of different ECG signal classification results based on the GPU-accelerated neural network model.

Acc, Se, Sp, and PR of the ECG signal S and V classification based on the GPU-accelerated neural network model were compared (Figure 9). Acc, Se, Sp, and PR of V were 99.03%, 89.17%, 98.92%, and 93.18% respectively. Acc, Se, Sp, and PR of S were 99.54%, 86.22%, 99.74%, and 92.56%, respectively. Figure 9 shows the comparison of V and S classification results based on GPU-accelerated neural network model.

The results of GRNN classification were compared with those of probabilistic neural network (PNN), particle swarm optimization algorithm (PSO), conditional random field (CRF), dynamic Bayesian network (DBN), and Kalman filter algorithms. The GRNN classification accuracy was up to 98%.  Figure 10 is the comparison of classification accuracy of different types of ECG signals by different algorithms.

### 3.1. Statistics of CPHD Prevalence

Statistics on the prevalence of CPHD in Figure 11 showed that a total of 1,935 COPD patients (19%) were diagnosed with CPHD, including 1,409 males (72.82%) and 526 females (36.24%). Figure 11 shows the statistics of CPHD prevalence.

### 3.2. Statistical Results of Various Parameters of CPHD Confirmed by ECG Diagnostic Criteria

Statistics on the proportion of patients under different parameters of the ECG of CPHD patients are shown in Figure 12. Of CPHD patients, the highest number of patients with Rv1 + Sv5 > 1.05 mV was 1,350 (69.77%), followed by 1,180 (60.98%) with V5R/S ≤ 1. At least 427 patients (22.07%) had V1∼3 of Qs, Qr, and qr. Figure 12 shows CPHD ECG parameter statistical results.

### 3.3. CPHD Distribution Statistics

The distribution of CPHD patients at different altitudes was statistically analyzed. The prevalence of CPHD patients decreased with the increase of altitude. The highest prevalence of CPHD was 64.60% at the altitude of 1,900–2,499 m and only 2.43% at the altitude of ≥3,500 m.  Figure 13 shows the distribution of CPHD patients at different altitudes.

The distribution of patients with CPHD at different ages was statistically analyzed. The prevalence of CPHD patients increased first and then decreased with the increase of patients' age. The highest prevalence of CPHD was 63.77% at the age of 61–70, and the lowest prevalence was only 0.26% at the age of 15∼20.  Figure 14 shows the distribution of CPHD patients at different ages.

The results showed that the processing time of ECG signals using the GPU neural network model was shortened by 20.2 times compared with that of the CPU. The calculation speed of the neural network model using GPU was dramatically improved. The reason was that the GPU's data cache was mainly embodied in a read-only form, which eliminated the access instructions of the video memory, thereby saving the video memory bandwidth [18]. In addition, GPU reduced the logic control unit and cache in the data processing process, thereby improving computational efficiency [19]. This was consistent with the findings of Fan et al. [20]. It was also found that the running time of the program using shared memory was about 4.8 times shorter than that of the program not using shared memory. The reason was that after shared memory was used, the average amount of computation dropped notably for a block. Moreover, the buffering of shared memory was performed on GPU, which further improved its computing speed. For the same number of ECG signals, CPU processing time was the longest, GTX780Ti processing time was the shortest, and GTX780Ti running time was about 15 times shorter than that of CPU. It was dramatically shorter than the running time of the openMP program proposed by Shikder et al. [21]. The result of ECG signal classification based on the GPU-accelerated neural network model indicated that the highest accuracy of detecting N reached 98.06%, which may be caused by the unobvious signals of the S, V, and F types of ECG or the too specificity of the N types of ECG signals. The classification accuracy of GRNN was up to 98%, and its classification accuracy was dramatically higher than the 95% classification accuracy of Celin et al. [22]. It showed that the neural network model based on GPU acceleration improved the accuracy of ECG signal classification.

The results revealed that the prevalence of CPHD was 19%. Bernocchi et al. [23] pointed out that the prevalence of CPHD in COPD patients was 18.9%. Moreover, the results of Sessa et al. [24] pointed out that the incidence of CPHD in COPD patients was 12.5%. The results of this article were greatly higher than those of these studies. The reason was that the patients in this study were in the plateau area, and the patients in these studies were distributed in the plain. Fors et al. [25] pointed out that the incidence of CPHD in COPD patients was 22.8%, which was similar to the results of this study. COPD patients in high-altitude areas had CPHD due to high-altitude hypoxia. The highest prevalence of CPHD was 64.60% when the altitude was 1,900–2,499 m, and the prevalence was only 2.43% when the altitude was ≥3,500 m. The research results of Roversi and Fabbri [26] suggested that the number of patients who died of CPHD in the plateau residents and lived for a long time at an altitude of more than 2,500 m increased notably, indicating that the occurrence of CPHD was correlated with altitude. The results of this study had certain deviations from them. The reason may be related to the population density, fresh air, and living habits in high-altitude areas. Residents living on plateaus greater than 2,500 m for a long time were mainly Tibetans, and the pulmonary artery pressure of Tibetans was similar to that of plain people [27]. Therefore, it was speculated that these people had adapted to the high-altitude and hypoxic environment. The highest prevalence of CPHD was 63.77% at the age of 61–70 years, and the lowest prevalence at the age of 15∼20 years was only 0.26%. It showed that the age range of 60–71 years old for patients COPD was correlated with a high incidence of CPHD, which was consistent with the results of Admon et al. [28].

## 4. Conclusion

Based on intelligent medical treatment and ECG signal big data, the factors of CPHD induced by plateau COPD are analyzed in this article. The results show that the GPU-based neural network model greatly improved the classification accuracy of ECG signals. Age and altitude were risk factors for CPHD induced by plateau COPD [29, 30]. However, there are still some shortcomings in this study. Biochemical indicators of plateau COPD were not analyzed in this study. In future work, we will further analyze the changes of biochemical indicators related to CPHD induced by plateau COPD to clarify these biochemical indicators. To sum up, the GPU-based neural network model improves the classification accuracy of ECG signals. Age and altitude are the risk factors of CPHD induced by COPD, which provides a reference basis for the prevention, diagnosis, and treatment of CPHD in the plateau area.

## Figures and Tables

**Figure 1:** ECG signal feature extraction based on GPU acceleration.

**Figure 2:** GPU-based GRNN algorithm.

**Figure 3:** Comparison of time-consuming feature extraction of different graphics cards.

**Figure 4:** Comparison of parallel parameter settings.

**Figure 5:** Comparison of the execution efficiency of the GRNN algorithm in GPU and CPU.

**Figure 6:** The operating efficiency of the GRNN algorithm in different hardware.

**Figure 7:** The results of different algorithms to locate QRS waves, (a) Quadratic spline wavelet, (b) Morlet wavelet, and (c) Symlet wavelet.

**Figure 8:** Comparison of different ECG signal classification results based on GPU-accelerated neural network model.

**Figure 9:** Comparison of V and S classification results based on GPU-accelerated neural network model.

**Figure 10:** Comparison of classification accuracy of different types of ECG signals by different algorithms.

**Figure 11:** Statistics of CPHD prevalence.

**Figure 12:** CPHD ECG parameter statistical results.

**Figure 13:** Distribution of CPHD patients at different altitudes.

**Figure 14:** Distribution of CPHD patients at different ages.

## Data Availability

The simulation experiment data used to support the findings of this study are available from the corresponding author upon request.
